# BA-GCA Net: Boundary-Aware Grid Contextual Attention Net in Osteosarcoma MRI Image Segmentation

**DOI:** 10.1155/2022/3881833

**Published:** 2022-07-30

**Authors:** Jia Wu, Zikang Liu, Fangfang Gou, Jun Zhu, Haoyu Tang, Xian Zhou, Wangping Xiong

**Affiliations:** ^1^School of Computer Science and Engineering, Central South University, Changsha 410083, China; ^2^Research Center for Artificial Intelligence, Monash University, Melbourne, Clayton VIC 3800, Australia; ^3^The First People's Hospital of Huaihua, Huaihua, Hunan, China; ^4^Collaborative Innovation Center for Medical Artificial Intelligence and Big Data Decision Making Assis-10 Tance, Hunan University of Medicine, Changsha, China; ^5^Jiangxi University of Chinese Medicine, Nanchang 330004, JiangXi, China

## Abstract

Osteosarcoma is one of the most common bone tumors that occurs in adolescents. Doctors often use magnetic resonance imaging (MRI) through biosensors to diagnose and predict osteosarcoma. However, a number of osteosarcoma MRI images have the problem of the tumor shape boundary being vague, complex, or irregular, which causes doctors to encounter difficulties in diagnosis and also makes some deep learning methods lose segmentation details as well as fail to locate the region of the osteosarcoma. In this article, we propose a novel boundary-aware grid contextual attention net (BA-GCA Net) to solve the problem of insufficient accuracy in osteosarcoma MRI image segmentation. First, a novel grid contextual attention (GCA) is designed to better capture the texture details of the tumor area. Then the statistical texture learning block (STLB) and the spatial transformer block (STB) are integrated into the network to improve its ability to extract statistical texture features and locate tumor areas. Over 80,000 MRI images of osteosarcoma from the Second Xiangya Hospital are adopted as a dataset for training, testing, and ablation studies. Results show that our proposed method achieves higher segmentation accuracy than existing methods with only a slight increase in the number of parameters and computational complexity.

## 1. Introduction

Osteosarcoma is the most common malignant bone tumor which occurs most frequently in children and adolescents between the ages of 10 and 30 years, with the highest incidence during the adolescent growth spurt [1]. In the past few years, neoadjuvant chemotherapy and biosensors have greatly developed, making the treatment of osteosarcoma easier. Nevertheless, without an early diagnosis, patients with advanced osteosarcoma will develop metastasis and recurrence disease, whose 5-year survival rate still keeps less than 20% [2, 3]. Therefore, how to clearly and accurately diagnose osteosarcoma has become the key to prevention and treatment.

Magnetic resonance imaging (MRI) can display the structure of soft tissue clearly and has higher contrast as well as resolution than other imaging methods [4], which makes the tumor area easier to distinguish. It is considered to be the best imaging method to evaluate the relationship between the primary osteosarcoma lesion and its surrounding areas [5]. Traditionally, the diagnosis of osteosarcoma is based on manual histopathological analysis with biosensors on MRI images by doctors. However, it has great disadvantages. In developing countries where the medical level is relatively backward, the doctor-patient ratio remains low, with each doctor handling the diagnosis and treatment of about 60 patients per day on average [6–8]. In addition, one patient will produce more than 600 MRI images during one diagnosis with biosensors, making analysis laborious and time-consuming [9–14]. To make matters worse, doctors' high-intensity work makes their manual judgments susceptible to inter- and intra-observer variations and results in inaccurate segmentation of osteosarcoma areas [15–17]. Furthermore, due to the heterogeneity of osteosarcoma [1], sophisticated diagnoses using MRI biosensors often require experienced radiologists, which is extraordinarily challenging for some developing countries with backward allocation of medical resources [18–20].

In order to solve the problems of manually segmenting lesions by doctors, researchers have designed a variety of automatic segmentation models and applied them to medical image segmentation to help doctors diagnose diseases and predict lesion areas, thus reducing the pressure on medical resources in developing countries and enabling diagnosis of diseases to achieve high accuracy at low computational costs. A fully convolutional network (FCN) [21] uses skip layers to achieve end-to-end and joint learning of semantic as well as location. It is the most classic model in medical image segmentation. U-Net [22] crops the output feature maps from shallow layers and concatenates them to the ones from deep layers to fuse and exploit the low-level and high-level features, improving the network's performance on neural structure and cell segmentation. In the specific field of osteosarcoma segmentation, [23] uses a recurrent convolutional neural network (RCNN) combining CNN and GRU and achieves better performance with a small number of histopathological osteosarcoma images. MSFCN [24] and MSRN [25] add multiple supervised structures to the network to promote learning and improve the overall osteosarcoma segmentation accuracy.

Considerable progress has been made in the research on osteosarcoma segmentation models. However, a few segmentation problems in MRI images using biosensors have unfortunately been overlooked: (i) The boundaries between osteosarcoma and normal tissues in some images are not clear enough and the lesion area is indistinguishable from other soft tissues. Therefore, the low-contrast boundaries may be blurred during convolution operations, resulting in segmentation failure. (ii) In transverse section images, the osteosarcoma area is often small, and the model is prone to spatial shift in the process of down-sampling and up-sampling, which leads to difficulty in localization and decrease in accuracy. (iii) Some osteosarcoma images have complicated and irregular shape boundaries, and the model cannot identify small gaps between osteosarcoma and normal tissues, causing the identification of the entire region as a lesion area and the loss of segmentation details. These problems contribute to poor performance on a number of difficult tasks with vague foreground-background boundaries or small and complex osteosarcoma regions, which have become a significant factor that affects the accuracy of segmentation.

In order to solve the problems mentioned above, we propose a novel boundary-aware grid contextual attention network (BA-GCA Net), which effectively improves the performance of the network on MRI images with blurred osteosarcoma boundaries and complex foreground structure. First, we propose a plug-and-play grid contextual attention structure. The structure splits the input feature map into patches, exploits the local contextual information to learn the positional features inside the image patches, and enhances the network's capability to capture the details of osteosarcoma boundaries and texture. For the problem that certain osteosarcoma MRI images using biosensors have intricate shape boundaries or fuzzy tumor texture, a statistical texture learning block (STLB) is integrated into the network. STLB learns the low-level features and applies them to the task. The texture enhancement module (TEM) in the STLB first enhances the texture in the low-level feature map and produces a clearer texture map, which is conducive to more accurate segmentation of the osteosarcoma region. Then the pyramid texture feature extraction module (PTFEM) is used in the STLB to further extract and utilize the enhanced texture. Due to the small tumor areas in some osteosarcoma MRI images, the subtle spatial shift of the prediction map will lead to poor segmentation performance. To this end, we use a spatial transformer block (STB) in the network to make it invariant to spatial shifts. STB localizes and regresses the input feature map, learns an affine transformation matrix, and applies the transformation to the feature map. It spatially adjusts the prediction map so that the positioning of osteosarcoma areas is more accurate.

In general, our contributions can be summarized as follows:

1. We propose a novel BA-GCA Net, which can better learn detailed features in the input image and fully exploit texture features in a spatially invariant way to improve the segmentation accuracy of osteosarcoma MRI images.
2. In order to pay more attention to local details in the input image, we propose a plug-and-play grid contextual attention (GCA) structure, which reshapes the image into patches and applies local and global contextual attention to them to enhance the perception of local details in osteosarcoma areas.
3. Inspired by U-Net, low-level features in the input image have rich texture details and therefore a statistical texture learning block (STLB) is used to learn texture features in the low-level feature map and utilize them in deeper layers of the network, improving the segmentation accuracy in tasks where the tumor area has blurred boundaries or small gaps.
4. To improve the model's ability in locating the osteosarcoma lesion area, we use an STB in the network to learn an affine transformation matrix and adjust the prediction map. Moreover, a boundary loss is designed in the loss function to facilitate STB to learn positional boundary information, which promotes the segmentation performance on images where the region of osteosarcoma is small.
5. Over 80,000 MRI images of osteosarcoma output by biosensors from the Second Xiangya Hospital are adopted as a dataset for experiments. Results show that our proposed method outperforms other models on accuracy with only a slight increase in the number of parameters and computational complexity compared with the backbone network and achieves a balance in terms of accuracy and computational efficiency, which is helpful to doctors in judging the osteosarcoma lesion area and reducing workload.

## 2. Related Works

### 2.1. Osteosarcoma Image Segmentation

Accurate diagnosis and prediction of osteosarcoma are the keys to increasing the survival rate of the patients and making precise follow-up treatment plans. Numerous researchers have studied in osteosarcoma image segmentation before. Reference [26] uses similarity mapping and slope value to analyze the time-intensity curves of regions of interest (ROI) and fuses the anatomic information of traditional MRI sequences with the numerical information of dynamic MRI sequences to obtain a better description of osteosarcoma regions. Reference [27] proposes a dynamic clustering algorithm DCHS based on Harmony Search (HS) and Fuzzy C-means (FCM) to automatically segment osteosarcoma MRI images, using a subset of Haralick texture features and pixel intensity values as a feature space to DCHS to delineate tumor volume, achieving a Dice measurement of an average of 0.72.

With the rapid development of deep learning and computer vision [28], a great number of deep learning-based models have been designed by researchers in the segmentation of osteosarcoma images as auxiliary diagnosis methods. Multiple supervised fully convolutional network (MSFCN) [24] adds supervision layers to the output layers of different sizes in the VGG model and uses the output information of the multiple supervision layers to produce the prediction map. Multiple supervised residual network (MSRN) [25] integrates residual structure into the network on the basis of multiple supervised structure, which improves the performance of a deep neural network on osteosarcoma image segmentation tasks. Wnet++ [29] uses two cascaded U-Nets and dense skip connections to realize automatic segmentation of tumor areas. In addition, Wnet++ adopts multi-scale input to alleviate information loss caused by down-sampling and introduces an attention mechanism to better represent tumor features, which increases the accuracy of segmentation. In osteosarcoma MRI image segmentation, there are often blurred foreground-background boundaries or small and complex segmentation regions. Therefore, the local semantic details and boundary information are of particular importance. Different from the above methods, we design BA-GCA Net, which embeds modules into the semantic segmentation framework to enhance the model's ability to extract rich local semantic, texture statistics, and boundary information and improves the model in performance on intricate segmentation tasks.

### 2.2. Boundary Prediction Enhancement Methods

In osteosarcoma MRI image segmentation, the prediction of boundaries is crucial to the model's performance. Previously, a great number of researchers in the field of medical image segmentation have devoted to solving the problem of segmentation boundaries [23–28]. Structure boundary preserving segmentation [30] obtains the structured boundary information of an image through a key point selection algorithm, a boundary preserving block, and a shape boundary-aware evaluator. BFP [31] utilizes a boundary-aware feature propagation module to transfer low-level boundary information. InverseForm [32] enables boundary loss function to learn spatial transformation distance through a pretrained inverse transformation network. Some other works [33–35] have improved the boundary loss function and achieved good results.

Unfortunately, the above methods neither take full advantage of the rich low-level statistical boundary texture features of the input image nor solve the problem of spatial shift of the prediction boundary that may exist in small osteosarcoma lesion areas. Unlike the above methods, we use a statistical texture learning block (STLB) [36] to quantify and count the low-level texture information output by the shallow layers in the network. Due to the segmentation of some small tumor areas in the osteosarcoma MRI images, spatial shifts may occur during down-sampling and up-sampling. Therefore, we integrate the STB [37] into the deep layer of the network to enhance the spatial transformation invariance. Combined with the boundary loss function, STB will automatically learn the spatial shift of the prediction map and adjust it adaptively.

### 2.3. Attention Mechanisms

Attention mechanism has been proved to raise the model's capability of giving more weight to useful features to improve semantic analysis and has achieved good results in a variety of computer vision tasks [38–42].

SENet [38] compresses feature maps in spatial dimension and generates a channel-wise attention. Based on SENet, CBAM [39] additionally introduces a spatial attention through channel pooling and large-scale convolution and has certain improvements in classification and detection. SANet [40] divides the segmentation task into two subtasks that are pixel-level prediction and pixel grouping and combines multi-scale prediction and pixel-grouping spatial attention to improve performance. OCR [41] learns the relationship between pixel and object region features based on coarse segmentation maps and enhances the description of pixel features. Coordinate attention (CA) [42] rethinks the attention mechanism and produces the attention map with positional information by compressing the spatial features of the image into attention weights in horizontal and vertical directions.

The above methods can extract image context in an efficient way, but cannot pay extra attention to the local details of the image that are indispensable for pixel-to-pixel osteosarcoma MRI image segmentation. Different from the above methods, our proposed grid contextual attention (GCA) combines local and global contextual attention, which can exploit the global contextual features of the feature map and learn local contextual features in the meantime.

## 3. Methods

As is mentioned above, the shortage of medical resources and the backward medical level in some developing countries make diagnosis of osteosarcoma more formidable. Moreover, the blurred and low-contrast tumor areas as well as small and intricate structural boundaries may lead to fuzzy or even wrong prediction of the lesion region from automatic segmentation models and influence clinical diagnoses. To this end, we add GCA, STLB, and STB to the network to reduce segmentation errors in osteosarcoma MRI images using biosensors while keeping the number of parameters and computational complexity at a low level to ensure low diagnostic cost. The overall structure of the network is shown in Figure 1.

For an osteosarcoma image generated by MRI biosensors, it is first fed into the backbone to extract high-level and low-level features. We integrate GCA at the top of the ResNet building blocks after the first two layers to improve the feature extraction ability of the model. The low-level features produced by the first two layers are fed into STLB to enhance and analyze texture statistics. The output of STLB is concatenated in channel dimension with the high-level features from the backbone added with GCA. Then the fused output is fed into STB to perform an affine transformation to the prediction map and produce the final output. Canny [43] operator is applied to the prediction result and ground truth to extract the boundaries. Segmentation loss and boundary loss are calculated using segmentation masks and boundaries, respectively, to form the compound loss function.

### 3.1. Grid Contextual Attention

In the pixel-wise osteosarcoma MRI image segmentation, understanding the local details in the image often helps in more accurate segmentation as well as less uncertain prediction. Therefore, we design a grid contextual attention (GCA) structure based on both local and global contextual features. The structure is shown in Figure 2.

For an input feature map *X* ∈ *R*^*C*×*H*×*W*^, its global contextual information is obtained by:

(1) $$\begin{array}{c} {\hat{A}}^{h}=\text{Excit}\left({\text{Avg}}_{w}\left(X\right)\right),\\ {\hat{A}}^{w}=\text{Excit}\left({\text{Avg}}_{h}\left(X\right)\right), \end{array}$$

where ${\hat{A}}^{h}\in R^{C\times H\times 1}$, ${\hat{A}}^{w}\in R^{C\times 1\times W}$, Avg_*h*_, and *Avg*_*w*_ denote average pooling of the feature map in height and width directions, respectively, and Excit denotes the activation transformation of the input as:

(2) $$\begin{array}{c} \text{Excit}\left(x\right)={\text{Conv}}_{\text{Sigmoid}}\left({\text{Conv}}_{\text{RELU}}\left(x\right)\right). \end{array}$$

In the part of local attention, GCA splits the feature map into patches, each of which is denoted as *P*_*i*,*j*_ ∈ *R*^*C*×*P*_*h*_×*P*_*w*_^, where *P*_*h*_ and *P*_*w*_ represent the patch size in height and width directions and *i* ∈ {1,2,…, (*H*/*P*_*h*_)}, *j* ∈ {1,2,…, (*W*/*P*_*w*_)}.

Each patch *P*_*i*,*j*_ is passed through average pooling in the width and the height directions respectively to get local attention *A*_*i*,*j*_^*h*^ ∈ *R*^*C*×*P*_*h*_×1^ and *A*_*i*,*j*_^*w*^ ∈ *R*^*C*×1×*P*_*w*_^. Then the patches are concatenated by:

(3) $$\begin{array}{c} A_{j}^{h}=\text{Concat}\left(A_{1,j}^{h},A_{2,j}^{h},\ldots ,A_{H/P_{h},j}^{h}\right),\\ A_{i}^{w}=\text{Concat}\left(A_{i,1}^{w},A_{i,2}^{w},\ldots ,A_{i,W/P_{w}}^{w}\right), \end{array}$$

where *i* ∈ {1,2,…, (*H*/*P*_*h*_)}, *j* ∈ {1,2,…, (*W*/*P*_*w*_)}, *A*_*j*_^*h*^ ∈ *R*^*C*×*H*×1^, and *A*_*i*_^*w*^ ∈ *R*^*C*×1×*W*^.

In order to enable localized patches to get global contextual information, each *A*_*j*_^*h*^ and *A*_*i*_^*w*^ are performed element-wise product with ${\hat{A}}^{h}$ and ${\hat{A}}^{w}$, respectively, to get ${\tilde{A}}_{j}^{h}$ and ${\tilde{A}}_{i}^{w}$.

After getting the global contextual information, compression and expansion are applied to ${\tilde{A}}_{j}^{h}$ and ${\tilde{A}}_{i}^{w}$, where compression uses a shared *Conv*_*Norm*−*RELU*_ to fuse attention maps in height and width directions and expansion applies Conv_Sigmoid_ to ${\tilde{A}}_{j}^{h}$ and ${\tilde{A}}_{i}^{w}$ separately to extract contextual features. Then ${\tilde{A}}_{j}^{h}$ and ${\tilde{A}}_{i}^{w}$ are divided into patches again to obtain ${\tilde{A}}_{i,j}^{h}$ and ${\tilde{A}}_{i,j}^{w}$, which are subsequently multiplied to get the attention maps *A*_*i*,*j*_^*m*^ ∈ *R*^*C*×*P*_*h*_×*P*_*w*_^. Specifically, *A*_*i*,*j*_^*m*^ is written as:

(4) $$\begin{array}{c} A_{i,j}^{m}={\tilde{A}}_{i,j}^{h}\times {\tilde{A}}_{i,j}^{w}, \end{array}$$

where × denotes matrix multiplication in spatial dimension.

Finally, *A*_*i*,*j*_^*m*^ and *P*_*i*,*j*_ are applied element-wise product to get the reweighted patches and the patches are concatenated, obtaining the output feature map *X*_out_ ∈ *R*^*C*×*H*×*W*^.

Compared with coordinate attention (CA) [42], GCA can better learn the local detailed features in the osteosarcoma MRI images while maintaining the global semantic features, which improves the segmentation accuracy in some blurred tumor images. In addition, to flexibly adjust the patch size and compensate for the loss of information between patches by using different patch sizes, padding-crop operation is designed in GCA. Through adaptive padding, the input feature map can be divided into patches of any size and be cropped back to the original input size after the attention operation.

### 3.2. Statistical Texture Learning Block

In osteosarcoma segmentation tasks, the rich contextual information contained in low-level features plays a crucial role in segmentation performance. To solve the problem of blurred boundaries as well as complex and irregular tumor shapes in osteosarcoma MRI images using biosensors, we use statistical texture learning block (STLB) [36] to fully exploit and utilize the texture features and combine the rich low-level features with the high-level features in the deeper layer of the network.

SFNet can combine low-level and high-level features with semantic flow. At the same time, STLB can explore the statistical features of osteosarcoma image texture [44, 45]. It not only learns the structural texture information, but also learns the global statistical information of the image, which is helpful for osteosarcoma segmentation. In this section, the 1d and 2d quantization and counting operator (QCO) are first introduced for statistical description of the texture information. Then two modules in STLB are introduced: the texture enhancement module (TEM) based on 1d-QCO to enhance the osteosarcoma texture features and the pyramid texture feature extraction module (PTFEM) based on 2d-QCO to further exploit the texture features.

#### 3.2.1. 1d-QCO

The structure of 1d-QCO is shown in Figure 3.

For an input feature map *X* ∈ *R*^*C*×*H*×*W*^, 1d-QCO applies global average pooling to *X* to get the average feature *a* ∈ *R*^*C*×1×1^. Then the cosine similarity between each pixel *X*_*i*,*j*_ in *X* and *a* is calculated to get *S* ∈ *R*^1×*H*×*W*^, where *i* ∈ {1,2,…, *H*} and *j* ∈ {1,2,…, *W*}. Each position *S*_*i*,*j*_ is denoted as:

(5) $$\begin{array}{c} S_{i,j}=\frac{a\cdot X_{i,j}}{{\left\|a\right\|}_{2}\cdot {\left\|X_{i,j}\right\|}_{2}}. \end{array}$$

Then *S* is reshaped to *S* ∈ *R*^*HW*^ and quantized to obtain the *N* levels *L*=[*L*_1_, *L*_2_,…, *L*_*N*_]. The nth level *L*_*n*_ is written as:

(6) $$\begin{array}{c} L_{n}=\frac{n}{N}\left(\text{max}\left(S\right)-\text{min}\left(S\right)\right)+\text{min}\left(S\right), \end{array}$$

where *N* is a hyperparameter and *n* ∈ {1,2,…, *N*}.

For the similarity *S*_*i*_ ∈ *R* of each pixel in the feature map, we encode it to *E*^*i*^ ∈ *R*^*N*^, where *i* ∈ {1,2,…, *HW*} and each dimension *n* ∈ {1,2,…, *N*} of *E*_*i*_ is calculated by:

(7) $$\begin{array}{c} E_{i,n}=\left\{\begin{array}{cc} 1-\left|L_{n}-S_{i},\right| & -\frac{0.5}{N}\leq L_{n}-S_{i}<\frac{0.5}{N},\\ 0, & \text{other.} \end{array}\right. \end{array}$$

The encoding map *E* ∈ *R*^*N*×*HW*^ consists of each pixel's encoded value. Compared with one-hot encoding or argmax operation, the quantization encoding is smoother and robust to gradient vanishing.

1d-QCO then applies counting operation to the encoding map *E* to get the counting map *M* ∈ *R*^*N*×2^. Concretely, *M* is calculated by:

(8) $$\begin{array}{c} M=\text{Concat}\left(L,\frac{\sum_{i=1}^{HW}E_{i,n}}{\sum_{n=1}^{N}\sum_{i=1}^{HW}E_{i,n}}\right), \end{array}$$

where Concat denotes concatenate operation in channel dimension.

Thereafter, the average feature *a* is up-sampled to *a* ∈ *R*^*N*×*C*^ and concatenated to the up-sampled *M* to produce *P* ∈ *R*^*N*×*C*_1_^, which is calculated by:

(9) $$\begin{array}{c} P=\text{Concat}\left(\text{Up}\left(M\right),a\right). \end{array}$$

The output of 1d-QCO includes the encoding map *E* as well as the statistical texture information *P* of osteosarcoma.

#### 3.2.2. 2d-QCO

1d-QCO contains the statistical texture features of the osteosarcoma images. However, it cannot learn positional relationships between pixels. Therefore, a 2d-QCO is proposed.

Similar to 1d-QCO, 2d-QCO calculates cosine similarity and level encoding of the input feature map *X* ∈ *R*^*C*×*H*×*W*^ to get the encoding map *E* ∈ *R*^*N*×*HW*^ and quantization levels *L*. Then *E* is reshaped to *E* ∈ *R*^*N*×1×*H*×*W*^. For the encoding of each adjacent pixel pair *E*_*i*,*j*_ ∈ *R*^*N*×1^ and *E*_*i*,*j*+1_ ∈ *R*^*N*×1^, the encoded value ${\hat{E}}_{i,j}\in R^{N\times N}$ that carries adjacent information is calculated by:

(10) $$\begin{array}{c} {\hat{E}}_{i,j}=E_{i,j}\times E_{i,j+1}^{T}, \end{array}$$

where *T* and × denote matrix transpose and multiplication, respectively. Then we get the encoding map $\hat{E}\in R^{N\times N\times H\times W}$ that contains adjacent features of the input.

In the counting process, the counting map *M* ∈ *R*^*N*×*N*×3^ is produced by:

(11) $$\begin{array}{c} M=\text{Concat}\left(\hat{L},\frac{\sum_{i=1}^{H}\sum_{j=1}^{W}{\hat{E}}_{m,n,i,j}}{\sum_{m=1}^{N}\sum_{n=1}^{N}\sum_{i=1}^{H}\sum_{j=1}^{W}{\hat{E}}_{m,n,i,j}}\right), \end{array}$$

where $\hat{L}\in R^{N\times N\times 2}$ represents the pairwise combination of all the quantization levels and ${\hat{L}}_{m,n}=\left[L_{m},L_{n}\right]$.

In 2d-QCO, the average feature is written as *a* ∈ *R*^*N*×*N*×*C*^ and the final output *P* ∈ *R*^*N*×*N*×*C*_1_^ is obtained by:

(12) $$\begin{array}{c} P=\text{Concat}\left(\text{Up}\left(M\right),a\right). \end{array}$$

#### 3.2.3. Texture Enhancement Module

The low-level texture such as structural boundaries in osteosarcoma images are often blurred and of low contrast. To this end, a texture enhancement module (TEM) is employed to sharpening the structural texture and make the low-level features easier to learn. The structure of TEM is shown in Figure 4.

Inspired by the histogram quantization method in traditional image processing algorithms, the statistical information in each quantization level is treated as a node in the graph adjacency matrix. Unlike the traditional method of defining a diagonal matrix artificially, TEM uses graph reasoning to construct the adjacency matrix and reconstruct the quantization level *L* to get *L*′. Concretely, the process can be written as:

(13) $$\begin{array}{c} G=\text{Softmax}\left(\text{Conv}\left(P^{T}\right)\times \text{Conv}\left(P\right)\right),\\ L^{\prime }=\text{Conv}\left(P\right)\times G. \end{array}$$

Finally, the output *O* ∈ *R*^*C*_2_×*H*×*W*^ is obtained using the reconstructed quantization levels *L*′ and the encoding map *E*. *O* ∈ *R*^*C*_2_×*H*×*W*^ is denoted as:

(14) $$\begin{array}{c} O=\text{Reshape}\left(L^{\prime }\times E\right), \end{array}$$

where Reshape represents reshaping the output to *O* ∈ *R*^*C*_2_×*H*×*W*^.

#### 3.2.4. Pyramid Texture Feature Extraction Module

The features of statistical texture in osteosarcoma MRI images are effectively enhanced through TEM. Then a pyramid texture feature extraction module (PTFEM) is proposed to extract and exploit rich texture features of the boundaries. The structure of PTFEM is shown in Figure 5.

Inspired by the conventional gray-level co-occurrence matrix algorithm, the input feature map of osteosarcoma is first passed through 2d-QCO to get the statistical co-occurrent features *P* ∈ *R*^*C*×*N*×*N*^ and then the texture features *T* ∈ *R*^*C*′^ is calculated using a MLP and a level-wise average operation. Specifically, the process is denoted as:

(15) $$\begin{array}{c} P^{\prime }=\text{MLP}\left(P\right),\;P^{\prime }\in R^{C^{\prime }\times N\times N},\\ T=\frac{\sum_{m=1}^{N}\sum_{n=1}^{N}P_{k,m,n}^{\prime }}{N\times N},\;k\in \left\{1,2,\ldots ,C^{\prime }\right\}. \end{array}$$

Some previous works such as FPN [46] and DeepLabV3+ [47] found that the employment of multi-scale structure can improve the model's performance. Inspired by these works, PTFEM integrates 2d-QCO with different scales into the structure to better extract and utilize the osteosarcoma texture features.

### 3.3. Spatial Transformer Block

Due to the small and complicated osteosarcoma lesion areas in some MRI images produced by biosensors, even a slight spatial shift of the prediction map can produce poor results, which in turn lead to wrong diagnosis. To this end, we use an STB [37] to make the backbone invariant to spatial transformation and more robust to the osteosarcoma images with small and intricate tumor regions.

For the high-resolution segmentation map of osteosarcoma, we assume that the error of the map to the ground truth can be reduced by homography transformation. Therefore, we use STB to learn this spatial transformation. The structure of STB is shown in Figure 6.

For an input feature map *X* ∈ *R*^*C*×*H*×*W*^, STB uses a set of down-sampling convolutions *F*_down−sample_ and fully connected layers *F*_regression_ to produce an affine transformation matrix *M*_affine_ ∈ *R*^2×3^. Concretely, *M*_affine_ is denoted as:

(16) $$\begin{array}{c} M_{\text{affine}}=F_{\text{regression}}\left(F_{\text{down}-\text{sample}}\left(X\right)\right). \end{array}$$

Simultaneously, the input feature map is applied a 1 × 1 convolution as well as a softmax activation in another branch to get the initial prediction map pred ∈ *R*^2×*H*×*W*^, which can be described as:

(17) $$\begin{array}{c} \text{pred}=\text{Softmax}\left(\text{Conv}\left(X\right)\right). \end{array}$$

We denote the affine matrix as $M_{\text{affine}}=\left[\begin{array}{ccc} a_{11} & a_{12} & a_{13}\\ a_{21} & a_{22} & a_{23} \end{array}\right]$. For the coordinates (*x*_*n*_^*s*^, *y*_*n*_^*s*^) of each pixel in the initial prediction map pred and the coordinates (*x*_*n*_^*t*^, *y*_*n*_^*t*^) of each pixel in the final prediction map pred′ ∈ *R*^2×*H*×*W*^, where *n* ∈ {1,2,…, *HW*}, the affine transformation is defined as:

(18) $$\begin{array}{c} \left(\begin{array}{c} x_{n}^{s}\\ y_{n}^{s} \end{array}\right)=M_{\text{affine}}\left(\begin{array}{c} x_{n}^{t}\\ y_{n}^{t}\\ 1 \end{array}\right)=\left[\begin{array}{ccc} a_{11} & a_{12} & a_{13}\\ a_{21} & a_{22} & a_{23} \end{array}\right]\left(\begin{array}{c} x_{n}^{t}\\ y_{n}^{t}\\ 1 \end{array}\right). \end{array}$$

In order to apply spatial transformation to the initial prediction map, STB samples each (*x*_*n*_^*s*^, *y*_*n*_^*s*^) to obtain the final output pred′. Specifically, the process can be represented as:

(19) $$\begin{array}{c} {\text{pred}}_{c,n}^{\prime }=\sum_{i=1}^{H}\sum_{j=1}^{W}{\text{pred}}_{c,i,j}\times I\left(x_{n}^{s}-j;\Phi_{x}\right)\times I\left(y_{n}^{s}-i;\Phi_{y}\right), \end{array}$$

where *I* denotes to bilinear interpolation, Φ_*x*_ and Φ_*y*_ denote sampling parameters, and *c* ∈ {1,2,…, *C*} represents the channel index of the feature map.

### 3.4. Compound Loss Function

To improve both the prediction accuracy and the boundary perception ability of the model for osteosarcoma, we design a compound loss function based on focal loss [48]. The loss function consists of a segmentation loss as well as a boundary loss.

#### 3.4.1. Weighted Segmentation Focal Loss

For the prediction map *y*_pred_ and the ground truth *y*_*gt*_, the weighted segmentation focal loss is defined as:

(20) $$\begin{array}{c} FL_{\text{seg}}=-\alpha y_{gt}{\left(1-y_{\text{pred}}\right)}^{\gamma }\log\left(y_{\text{pred}}\right)\left(1-\alpha \right)\left(1-y_{gt}\right)y_{\text{pred}}^{\gamma }\log\left(1-y_{\text{pred}}\right), \end{array}$$

where *α* and *γ* represent the balance weight and the exponential hyperparameter, respectively.

#### 3.4.2. Weighted Boundary Focal Loss

In osteosarcoma MRI image segmentation, the boundary plays an essential role in improving the segmentation performance. Therefore, we introduce a weighted boundary focal loss to facilitate the model to learn boundary information.

First, the segmentation head and the ground truth are applied Canny [43] operator to produce the prediction and ground truth boundary *b*_pred_ and *b*_*gt*_. Then we perform edge sharpening on the normalized *b*_*gt*_ with a threshold of 0.5 and obtain a clear ground truth boundary *b*_*gt*_′. The weighted boundary focal loss is calculated using *b*_pred_ and *b*_*gt*_′ as:

(21) $$\begin{array}{c} FL_{\text{boundary}}=-\alpha b_{gt}^{\prime }{\left(1-b_{\text{pred}}\right)}^{\gamma }\text{log}\left(b_{\text{pred}}\right)-\left(1-\alpha \right)\left(1-b_{gt}^{\prime }\right)b_{\text{pred}}^{\gamma }\text{log}\left(1-b_{\text{pred}}\right). \end{array}$$

The compound loss function is defined as:

(22) $$\begin{array}{c} \text{Loss}=FL_{\text{seg}}+\beta FL_{\text{boundary}}, \end{array}$$

where *β* is the hyperparameter of weight. After experiments, one of the suitable values of *β* is 0.2, which is used in this article.

The compound loss function enables the model aware of the boundaries of osteosarcoma and also promotes STB to learn the spatial transformation between the prediction output and the ground truth, which in turn makes the model more robust to tumor segmentation. BA-GCA Net is trained in combination of compound loss function, enhancing the model's ability to boundary localization. As a method to assist doctors in diagnosis, it reduces the doctors' workload and improves the accuracy of diagnosis.

## 4. Experiments

In this section, we employ over 80,000 MRI images of osteosarcoma output by biosensors from 204 cases as the dataset for experiments to evaluate the model and perform ablation studies, which are provided by the Ministry of Education Mobile Health Information-China Mobile Joint Laboratory and the Second Xiangya Hospital of Central South University [49].

### 4.1. Dataset

We have collected statistics about patients and the results are shown in Table 1. We randomly select 80% of the images for training and the remaining 20% for evaluation. To be specific, there are a total of 204 case samples, of which 164 are in the training set and 40 are in the test set.

Due to the confidentiality of data between hospitals and the privacy of patients, the dataset is relatively hard to obtain, which leads to the overfitting problem of the model. To promote the robustness of the model to new data, we perform data augmentation on the training set. We rotate the images at 3 angles (0, 90, and 180), flip the image on different axes (no flip, up-down, and left-right), perform Gaussian blurring, add Gaussian noise (using different variances), and apply salt and pepper noise (using different proportions) to augment the training set.

### 4.2. Evaluation Metrics

In order to evaluate the performance of the model on osteosarcoma MRI image segmentation, in this section, we introduce accuracy, precision, recall, *F*1-score, Dice similarity coefficient (DSC) [50], and Intersection of Union (IOU) as the evaluation metrics and the confusion matrix with true positives (TP), false positives (FP), true negatives (TN), and false negatives (FN) to explain the performance of the model [51]. The evaluation metrics are defined as follows:

Accuracy (Acc) is used to evaluate the proportion of the model's right prediction and it is denoted as [52]:

(23) $$\begin{array}{c} \text{accuracy}=\frac{\text{TP}+\text{TN}}{\text{TP}+\text{TN}+\text{FP}+\text{FN}}. \end{array}$$

precision (Pre) is to calculate the percentage of true osteosarcoma areas among the prediction areas [53]. Precision can be written as:

(24) $$\begin{array}{c} \text{precision}=\frac{\text{TP}}{\text{TP}+\text{FP}}. \end{array}$$

recall (Rec) evaluates the percentage of the prediction osteosarcoma areas among the true areas [54]. Concretely, recall is denoted as:

(25) $$\begin{array}{c} \text{recall}=\frac{\text{TP}}{\text{TP}+\text{FN}}. \end{array}$$

*F*1 indicates the robustness of segmentation and is defined as [55]:

(26) $$\begin{array}{c} F1=\frac{2*\text{precision}*\text{recall}}{\text{precision}+\text{recall}}. \end{array}$$

For a simpler description of DSC as well as IOU, we denote the prediction of tumor area as *y*_pred_ and the ground truth as *y*_*gt*_.

DSC represents the similarity between *y*_pred_ and *y*_*gt*_. DSC can be written as

(27) $$\begin{array}{c} \text{DSC}=\frac{2\left|y_{\text{pred}}\cap y_{gt}\right|}{\left|y_{\text{pred}}\right|+\left|y_{gt}\right|}. \end{array}$$

IOU measures the degree of overlap between the model's prediction map and the ground truth and it is denoted as [56]

(28) $$\begin{array}{c} \text{IOU}=\frac{y_{\text{pred}}\cap y_{gt}}{y_{\text{pred}}\cup y_{gt}}. \end{array}$$

Furthermore, we adopt #params as the number of parameters of the model and use floating point operations (FLOPs) to evaluate the computational complexity [57, 58].

#### 4.2.1. Training Details

The Dilated ResNet-D-22(DRN-D-22) [52] is chosen as the backbone and BA-GCA Net is designed based on it. Note that osteosarcoma MRI images often have large individual differences, and the relationship between pixels in one image plays a more crucial role than that among images. To this end, we replace batch norm in the backbone to layer norm. Other hyperparameters of the model are shown in Table 2.

### 4.3. Comparison with Other Methods

Figure 7 shows the performance of each model on osteosarcoma MRI image segmentation. Column (A) represents the original image, columns (B)-(K) are the prediction output of each model, and column (L) is the ground truth. Note that BA-GCA Net outperforms other models in some difficult tasks, such as the second image that has low contrast and blurred boundaries, the fourth image of transverse section with small and complicated tumor area, and the last image that contains small gaps in the region of osteosarcoma. Results show that our proposed BA-GCA Net has better performance than some latest methods such as DeepLabV3 and UNet++ in capturing boundary details and recognizing blurred osteosarcoma lesion areas. Furthermore, BA-GCA Net is more robust to segmentation and DSC of its prediction remains above 0.93 in difficult segmentation tasks. Compared with other models, BA-GCA Net shows an advantage in processing the low-contrast and complex osteosarcoma images and localizing the small tumor regions, which is helpful for clinical diagnosis.

The quantitative evaluation results of BA-GCA Net and other comparative models on the test set are shown in Table 3. From the results we know that BA-GCA Net achieves higher precision, *F*1-score, DSC, and IOU than latest methods, which means our proposed method performs better overall on the test set. By integrating GCA, STLB, and STB into the backbone, the DSC of the model has increased by 0.004, 0.003, and 0.011 and the IOU of the model has increased by 0.023, 0.007, and 0.007, respectively. It is proved that the three blocks effectively strengthen the backbone with an increase of DSC by 0.018 and increase of IOU by 0.037. More detailed analysis will be introduced in the Ablation Study section.

The relationship between the number of parameters and DSC of different models is shown in Figure 8. It shows that BA-GCA Net achieves the highest DSC among all the models. Compared with UNet++, BA-GCA Net has a 0.019 higher DSC with only a slight increase in the number of parameters by 0.19 M. Moreover, BA-GCA Net outperforms the DRN added with coordinate attention (CA) [42] on DSC increasing by 0.017 and has only an increase in the number of parameters by 1.82 M.

The comparison of FLOPs and DSC between models is shown in Figure 9. We can know from the results that the computational cost of our proposed method is higher than DRN added with CA by 72.49GFLOPs and lower than U-Net by 10.46GFLOPs, which achieves a good balance between the accuracy and the computational complexity.

## 5. Ablation Study

In this section, ablation studies on the three blocks are introduced respectively in order to better analyze the role as well as the necessity of each block in BA-GCA Net. By comparing the performance of the model with and without the block, and visualizing the outputs in the middle layers, we can check out whether a block plays the role as expected.

### 5.1. Ablation of GCA

Attention mechanism is able to calibrate the input feature map so that the model can focus on the regions of interest. To illustrate that GCA can learn this calibration more precisely, in this section, we employ Seg-Grad-CAM [61] to visualize GCA as well as CA [42]. By summing the partial derivatives of the output target region with respect to the feature maps before and after the last GCA block (or CA block), respectively, and taking the mean of the derivatives for each channel as the weight of the feature map, we can visualize the influence of the attention block. The visualization results of GCA and CA are shown in Figure 10. Yellow and red indicate that the model gives higher weight to the region, while green and blue are the opposite. The visualization only computes the partial derivatives of the osteosarcoma region in the ground truth. The images show that GCA is more sensitive to the osteosarcoma areas and locates the tumor regions more precisely. Compared with CA, our proposed structure can better observe the tumor details and calibrate the feature map.

The DSC and IOU indicators and number of parameters of DRN, DRN with CA, and DRN with GCA are shown in Table 4, respectively. Compared with CA, the number of parameters of GCA is only 0.05 M more, but the DSC and IOU have increased by 0.003 and 0.015, respectively.

### 5.2. Ablation of STLB

STLB provides an effective method for better extracting and utilizing low-level texture features of the input images. A key role in STLB is the texture enhancement module (TEM). To analyze what TEM learns during training, we visualize the input and output feature maps of the TEM, mapping the grayscale values to colors from blue to red, which is shown in Figure 11. Note that through quantization, counting, and texture enhancement, the boundaries and some texture of the tissues such as bones, muscles, and osteosarcomas are exploited and sharpened to produce clearer feature maps, which is helpful for PTFEM to extract the spatial correlation features between pixels.

Table 5 shows the changes of DSC, IOU, and number of parameters of the model before and after adding STLB. Compared with DRN-D-22, the DRN added with STLB achieves an increase in DSC and IOU by 0.005 and 0.019, respectively, and the number of parameters increases by only 0.35 M. STLB enhances and utilizes the texture details and statistical features of osteosarcoma images, thereby improving the performance on low-contrast and blurred tumor segmentation tasks.

### 5.3. Ablation of STB

As is mentioned above, STB learns to perform affine transformation on the prediction map to better locate the tumor area. In this section, we examine the segmentation effect before and after affine transformation, as shown in Figure 12. Column (D) shows the comparison of boundaries before and after STB. Canny filter is used to extract the boundary. The red one is the output boundary before STB, and the blue one is the opposite. From the changes of DSC, we can conclude that STB performs beneficial spatial transformation on the input feature map, making the prediction area more accurate. By integrating STB into the model, the spatial shift and deformation caused by down-sampling and up-sampling are corrected, and the DSC and IOU has increased by 0.011 and 0.007, respectively.

## 6. Conclusion

In this article, we use a novel GCA, STLB, and STB to improve the model's segmentation performance on some difficult tasks such as complex osteosarcoma boundaries, small tumor areas, and low-contrast images produced by MRI biosensors. We propose a BA-GCA Net with the three blocks and employ over 80,000 MRI images of osteosarcoma from the Second Xiangya Hospital in China to train and test the model. In order to check out the function of each block, we conduct ablation studies. The visual analysis of the results helps us understand how each block works and its effectiveness. The test results show that out proposed BA-GCA Net achieves 0.927 DSC and 0.880 IOU, which is better than other existing models. The number of parameters and computational cost are only 19.88 M and 149.70GFLOPs, respectively, which means the model reaches a balance between accuracy and computational consumption. The model can assist doctors in judging the area of osteosarcoma at a relatively low cost, reduce the workload of doctors, and improve the efficiency of diagnosis.

In the future, in view of the difficulty in obtaining the clinical data of osteosarcoma, we will introduce few-shot learning into our method, so that the model can use fewer samples to obtain similar results. It will solve the problem of insufficient generalization of hospital self-trained models due to the data incompatibility between hospitals, improve the robustness of the model, and reduce training costs.

## Figures and Tables

**Figure 1:** The overall structure of BA-GCA Net.

**Figure 2:** The structure of grid contextual attention (GCA).

**Figure 3:** The structure of 1d-QCO.

**Figure 4:** The structure of the texture enhancement module.

**Figure 5:** The structure of pyramid texture feature extraction module.

**Figure 6:** The structure of spatial transformer block (STB).

**Figure 7:** The segmentation effects of models on some osteosarcoma MRI images.

**Figure 8:** Comparison of #params and DSC between models.

**Figure 9:** Comparison of FLOPs and DSC between models.

**Figure 10:** Visualization results of GCA and CA.

**Figure 11:** Visualization of feature maps before and after TEM.

**Figure 12:** Visualization of prediction boundaries before and after STB.

**Table 1:** Patient statistics.

Characteristics	Total	Training set	Test set
Age			
<15	48 (23.5%)	38 (23.2%)	10 (25.0%)
15–25	131 (64.2%)	107 (65.2%)	24 (60.0%)
>25	25 (12.3%)	19 (11.6%)	6 (15.0%)

Sex			
Female	92 (45.1%)	69 (42.1%)	23 (57.5%)
Male	112 (54.9%)	95 (57.9%)	17 (42.5%)

Marital status			
Married	32 (15.7%)	19 (11.6%)	13 (32.5%)
Unmarried	172 (84.3%)	145 (88.4%)	27 (67.5%)

SES			
Low SES	78 (38.2%)	66 (40.2%)	12 (30.0%)
High SES	126 (61.8%)	98 (59.8%)	28 (70.0%)

Surgery			
Yes	181 (88.8%)	146 (89.0%)	35 (87.5%)
No	23 (11.2%)	18 (11.0%)	5 (12.5%)

Grade			
Low grade	41 (20.1%)	15 (9.1%)	26 (65.0%)
High grade	163 (79.9%)	149 (90.9%)	14 (35.0%)

Location			
Axial	29 (14.2%)	21 (12.8%)	8 (20.0%)
Extremity	138 (67.7%)	109 (66.5%)	29 (72.5%)
Other	37 (18.1%)	34 (20.7%)	3 (7.5%)

**Table 2:** Hyperparameters of the model.

stage	Hyperparameter	Value
GCA block	Strategy	Residual

ST block	Weight	Zero
	Bias	[1, 0, 0, 0, 1, 0]
	Interpolation method	Bilinear

STL block	num_levels	128

Loss function	*α*	Based on ratios in batch
	*β*	0.2
	*γ*	1.25

Training	Initializer	kaiming_uniform
	Epochs	200
	Base learning rate	0.0001
	Optimizer	Adam
	Learning rate decay	(1 − (epoch/total_epochs))^0.9^
	Up-sampling	Bilinear

**Table 3:** Performance of models.

Model	Pre	Rec	F1	DSC	IOU	#params	FLOPs
FCN-16s [21]	0.922	0.882	0.900	0.859	0.824	134.3 M	190.35 G
FCN-8s [21]	0.892	0.914	0.902	0.875	0.831	134.3 M	190.08 G
MSFCN [24]	0.881	0.936	0.906	0.874	0.841	23.38 M	1524.34 G
MSRN [25]	0.893	0.945	0.918	0.887	0.853	14.27 M	1461.23 G
FPN [46]	0.914	0.924	0.919	0.888	0.852	48.20 M	141.45 G
U-Net [22]	0.922	0.924	0.923	0.892	0.867	17.26 M	160.16 G
OCR [41]	0.897	0.908	0.901	0.891	0.827	27.35 M	125.67 G
DeepLabV3 [4]	0.926	0.925	0.925	0.909	0.870	39.63 M	170.45 G
UNet++ [59]	0.924	0.924	0.924	0.908	0.868	18.16 M	165.23 G
SVM [60]	0.756	0.764	0.760	0.734	0.702	—	—
DRN [50]	0.916	0.922	0.917	0.909	0.843	17.66 M	76.93 G
DRN + CA [42]	0.918	0.923	0.919	0.910	0.851	18.06 M	77.21 G
Ours (DRN + GCA)	0.927	0.924	0.925	0.913	0.866	18.11 M	77.34 G
Ours (DRN + GCA + STLB)	0.925	0.934	0.929	0.916	0.873	18.47 M	82.67 G
Ours (DRN + GCA + STLB + STB)	0.938	0.937	0.937	0.927	0.880	19.88 M	149.70 G

**Table 4:** Performance of backbone with GCA and CA.

Model	param add (M)	#params (M)	DSC	IOU
DRN-D-22	—	17.66	0.909	0.843
+CA	+0.4	18.06	0.910 (+0.001)	0.851 (+0.008)
+GCA	+0.45	18.11	0.913 (+0.004)	0.866 (+0.023)

**Table 5:** Comparison of performance before and after using STLB.

Model	Param Add (M)	#params (M)	DSC	IOU
DRN-D-22	—	17.66	0.909	0.843
+STLB	+0.35	18.01	0.914 (+0.005)	0.862 (+0.019)

## Data Availability

The data used to support the findings of this study are currently under embargo while the research findings are commercialized. Requests for data, 12 months after publication of this article, will be considered by the corresponding author.
